The article "Association of ABO blood groups with ovarian reserve: a retrospective cohort study in Chinese Han women younger than 40 years with infertility" was published in 2022. Journal: J Ovarian Res.

# Association of ABO blood groups with ovarian reserve: a retrospective cohort study in Chinese Han women younger than 40 years with infertility

**DOI:** 10.1186/s13048-022-01075-0

**Published:** 2022-12-20

**Authors:** Xingyu Sun, Chenyu Sun, Muzi Meng, Ling Liu

**Affiliations:** 1 Department of Gynecology, The Affiliated Traditional Chinese Medicine Hospital of Southwest Medical University, Luzhou, 646000 Sichuan China; 2 Department of Reproductive Medicine Center, the Affiliated Hospital of Southwest Medical University, 25 Taiping Street, Luzhou, China; 3 AMITA Health Saint Joseph Hospital Chicago, 2900 N. Lake Shore Drive, Chicago, IL 60657 USA; 4 UK Program Site, American University of the Caribbean School of Medicine, Vernon Building Room 64, Sizer St, Preston, PR1 1JQ UK; 5 Bronxcare Health System, 1650 Grand Concourse, The Bronx, NY 10457 USA

**Keywords:** ABO blood type, Ovarian reserve, Infertility, Chinese Han women, Younger than 40 years

## Abstract

**Background:**

Ovarian reserve reflects both the quantity and quality of oocytes available for procreation and is affected by many known and unknown factors. ABO blood type is related to several infertility processes, but it is unclear whether and how ABO blood type affects ovarian reserve.

**Objective:**

The purpose of the study was to explore the correlation between ABO blood types and ovarian reserve in infertile Chinese Han women under 40 years of age undergoing the in vitro fertilization (IVF)/ intracytoplasmic sperm injection (ICSI)-embryo transfer (IVF/ICSI-ET) treatment.

**Methods:**

Women aged < 40 years who underwent IVF/ICSI-ET at our institution and had a documented ABO blood type were eligible for this study. In this study, patients were divided into two groups according to the diminished ovarian reserve (DOR) group (AMH < 1.1 ng/mL, AFC < 6) and the non-diminished ovarian reserve (non-DOR) group (AMH ≥ 1.1 ng/mL, AFC ≥ 6). The relationship between ovarian reserve and ABO blood group was determined by correlation analysis.

**Results:**

In this retrospective cohort study, clinical data were collected from 1690 Chinese Han women treated with IVF/ ICSI-ET in hospital records between April 2019 and March 2020 in the affiliated hospital of Southwest Medical University, located in Luzhou, China. The differences in age, duration of infertility, BMI, FSH, FSH / LH, and p (DOR vs non-DOR) for each parameter (DOR vs non-DOR) were statistically significant, and the differences in LH and E2 were not statistically significant. ABO blood groups were most prevalent in the DOR group with O (143, 34.8%) and A (122, 29.7%) and in the non-DOR group with A (428, 33.5%) and O (419, 32.8%). ABO blood groups were most prevalent in the DOR group with O (*n* = 57, 30.5%) and A (*n* = 54, 28.9%) and in the non-DOR group with A (*n* = 335, 34.0%) and O (*n* = 323, 32.8%) were the most frequent in the non-DOR group.

**Conclusions:**

In this retrospective cohort study, we confirmed the lack of a significant association between ABO blood type and ovarian reserve. Further studies are needed to clarify whether there is any prognostic correlation between ABO blood group and ovarian reserve in women undergoing IVF/ICSI-ET.

## Introduction

Infertility is a common concern for couples [1, 2]. Infertility is defined as the inability to conceive within 12 months of unprotected sexual intercourse [3]. About 15% of couples worldwide suffer from infertility [4]. In women, this disorder is associated with increasing age and may also be caused by various underlying pathophysiologic mechanisms [5]. In vitro fertilization (IVF) is a frequently used treatment method to achieve pregnancy [6]. The success rates of IVF are increased under conditions that response well to controlled ovarian stimulation (COS) [7]. In addition to improving obstetric outcomes, better diagnosis and treatment of these mechanisms could improve paternity and long-term health [8] and result in significant cost savings in fertility treatment [9].

Diminished ovarian reserve is defined by a decreased quantity or quality of ovarian follicles in women. It is a condition between normal reproductive physiology and premature ovarian insufficiency. Although the criteria for diminished ovarian reserve have not been defined and vary from region to region [10], it is basically characterized by an elevated serum follicle stimulating hormone level, decreased anti-Müllerian hormone level, and diminished antral follicle count on ultrasonography. Diminished ovarian reserve is often associated with poor ovarian stimulation response, high cancellation rate and significantly lower pregnancy rates in vitro fertilization cycles. Diminished ovarian reserve is characterized by poor fertility outcomes even with assisted reproductive techniques, which is a major challenge in reproductive medicine [11]. Poor response to ovarian stimulation usually indicates a reduced response to follicular stimulation, which results in a reduced number of retrieved oocytes [12]. ABO blood group is associated with several diseases [13], including cardiovascular disease (CVD) [14], as well as digestive system neoplasms (gastric and pancreatic cancer) [15] and ovarian cancer [16, 17].

There has been interest in the relationship between infertility and ABO blood groups. Many studies have investigated the association of ABO blood groups with diminished ovarian reserve (DOR), but have obtained contradictory results. An increase in live birth rates has been found for blood group B by Goldsammler et al. [18]. In subsequent studies, it has been found, however, that ABO blood group does not influence IVF pregnancy outcomes [19, 20]. In addition, these [21] and other [22] authors have demonstrated that the association between the ABO blood group and ovarian reserve, and showed that blood group O is more likely to have diminished ovarian reserve (DOR) It has been reported that antigen A may be a protective factor of ovarian reserve capacity and that type O blood decreases the risk of ovarian reserve capacity more than blood types A and AB. Moreover, a report by WebMD Health News [23], proposed that type O blood is associated with infertility. According to some studies, women with antigen B are more likely to develop DOR [24], and subsequent studies found that ABO blood group had no effect on ovarian reserve or ovarian response [25–30]. Lin et al. showed that Chinese women with blood type O had less diminished ovarian reserve than women with blood type B and AB, which were more frequently associated with diminished ovarian reserve, whereas blood type A was not associated with ovarian reserve [24]. Pereira et al. studied a subgroup of patients with diminished ovarian reserve and found no difference in response to ovarian stimulation [31].

To date, the relationship between ABO blood groups and ovarian reserve is complex and study findings are sometimes contradictory and therefore additional studies are necessary to reconcile these conflicting findings. Accordingly, in the present study, we sought to assess the potential association between ABO blood groups and ovarian reserve in a cohort of women undergoing IVF/ICSI-ET.

## Materials and methods

### Patient enrollment

A total of 1690 Chinese Han women diagnosed with infertility were included in this retrospective cohort study at the Reproductive Medicine Center of Affiliated Hospital of Southwest Medical University, Luzhou, Sichuan, from April 2019 to March 2020. Inclusion Criteria: (a) Ethnicity was Han. (b) No history of alcoholism, smoking, etc. (c) Both couples were chromosomally normal. (d) These infertile women were diagnosed with tubal factor infertility, including hydrosalpinx and proximal tubal obstruction. (e) Patients with clinical information. Exclusion Criteria: (a) Chromosomal abnormalities in one or both spouses. (b) Women with PCOS. Patients enrolled in the study were divided into two groups: diminished ovarian reserve (DOR) group (AMH < 1.1 ng/mL, AFC < 6) and non-diminished ovarian reserve (non-DOR) group (AMH ≥ 1.1 ng/mL, AFC ≥ 6) based on patients’ AMH and AFC. The flow chart and selection process of participants are detailed as shown in Fig. 1.

**Fig. 1:** The flow chart of this research

### Clinical tests

Clinical information included age, duration of infertility, BMI (Body mass index), follicle stimulating hormone(FSH), luteinizing hormone(LH), FSH/LH, estradiol(E_2_), progesterone (P), and ABO blood group. Serum levels of sex hormone were measured by using an automated chemiluminescence enzyme immunoassay analyzer (HISCL-5000, Sysmex, Kobe, Japan). The serum AMH level was measured by using the electrochemiluminescence immunoassay kit (ACCESS AMH; Beckman Coulter, Inc., Brea, CA, USA). Serum follicle stimulating hormone(FSH), luteinizing hormone(LH), FSH/LH, estradiol(E2), and progesterone(P) levels were measured between day 2 and day 5 of the menstrual cycle. Serum follicle stimulating hormone(FSH), luteinizing hormone(LH), FSH/LH, estradiol(E2), and progesterone(P) levels were measured between day 2 and day5 of the menstrual cycle. AFC (antral follicle count) was measured using transvaginal ultrasound (Philips Healthcare, Amsterdam, the Netherlands).

### Statistical analysis

Statistical results were expressed as median and interquartile range of non-normally distributed variables. The measured data were conducted using the Shapiro-Wilk (SW) normality test. The Mann-Whitney test was used to compare the two groups. Count data were expressed as percentages (%) and analyzed by the χ 2 test. Statistical Analysis SPSS 19.0 (Version 19.0; SPSS Inc., Chicago, IL, USA) statistical software was used for statistical processing. A *P*-value of < 0.05 was considered statistically significant.

## Results

### Basic information of patients of the DOR group and non-DOR group

The median age was higher in the DOR group than in the non-group (35 vs. 31), with a statistically significant difference (***P*** < 0.001). There were significant differences between the DOR and non-group in terms of duration of infertility, BMI, basal FSH, basal FSH/LH, and basal P (***P*** < 0.05). All statistical results are shown in Table 1.

**Table 1:** Comparison of general characteristics between the two groups for infertile women

	n	age (years)	Duration of infertility (years)	BMI (kg/m^2^)	FSH (mlU/mL)	LH (mlU/mL)	FSH/LH	E2 (pg/mL)	P (ng/mL)
DOR	411	35 (31-38)	4 (2-7)	22.38(20.40-24.22)	10.93(9.1-13.8)	3.39(2.28-4.63)	3.38(1.67-3.96)	42.26(32.74-64.06)	0.57(0.35-1.05)
non-DOR	1279	31 (28-34)	3 (2-6)	21.63(19.92-24.03)	8.74(7.03-10.68)	3.42(2.24-5.23)	2.63(1.67-3.96)	42.26(32.74-64.06)	0.66(0.40-1.16)
***z***		−12.796	−1.970	−3.135	−11.858	− 1.095	−7.325	−0.923	−3.072
***P***		<0.001	0.049	0.002	<0.001	0.273	<0.001	0.356	0.002

Data presented as a median and interquartile range; Continuous variables were compared using the Mann-Whitney test

*BMI* Body mass index, *P* Progesterone, *FSH* Follicle stimulating hormone, *LH* Luteinizing hormone, *E2* Estradiol

### Correlation analysis of basic parameters and ovarian reserve

Spearman correlation analysis revealed that serum AMH levels were correlated with age, duration of infertility, BMI, FSH, FSH/LH, and P, and AFC was correlated with age, FSH, and FSH/LH. Results are shown in Table 2.

**Table 2:** Correlation analysis of basic parameters and ovarian reserve

	Age (years)	Duration of infertility (years)	BMI (kg/m^**2**^)	FSH (mlU/mL)	FSH/LH	P (ng/mL)
**AMH(ng/mL)**						
**r**	−0.388	−0.050	− 0.052	−0.327	− 0.294	0.064
**P**	<0.001	0.04	0.031	<0.001	<0.001	0.008
**AFC**						
**r**	−0.221	−0.037	−0.042	− 0.222	−0.114	0.033
**P**	<0.001	0.128	0.081	<0.001	<0.001	0.178

Data presented as a median and interquartile range; Continuous variables were compared using the Mann-Whitney test

*BMI* Body mass index, *P* Progesterone, *FSH* Follicle stimulating hormone, *LH* Luteinizing hormone, *E2* Estradiol

### Relationship between the distribution of the ABO blood type and the ovarian reserve

As shown in Table 3, patients were divided into two groups based on AMH concentration and AFC, Subjects with AMH < 1.1 ng/mL and AFC < 6 were assigned to DOR group (*n* = 411), and those with AMH ≥ 1.1 ng/mL and AFC ≥ 6 were assigned to non-DOR (*n* = 1279). The proportions of blood type O (34.8% vs. 32.8%; *p* = 0.470) were higher in DOR group than non-DOR group. There were more patients with type O than other blood types in the DOR group aged less than 40 years (34.8%), whereas there were more patients with type A than other blood types in the non-DOR group (33.5%). Overall, blood type O was the most prevalent in the DOR group (34.8%), followed by blood type A (29.7%), blood type B (27.3%), and blood type AB (8.3%). In parallel, blood type A was the most prevalent (33.5%), followed by blood type O (32.8%), blood type B (24.1%), and blood type AB (9.7%) in the non-DOR group aged less than 40 years. There were no significant differences in the proportions of blood types between the groups (PO = 0.470, PA = 0.164, PB = 0.213, PAB = 0.436, respectively). The above results indicate that the blood type is not related to ovarian reserve. The detailed results are shown in Table 3.

**Table 3:** The distributions of ABO blood type in the DOR group and non-DOR. [(%)]

	n	ABO blood type			
		O	A	B	AB
DOR	411	143(34.8)	122(29.7)	112(27.3)	34(8.3)
non-DOR	1279	419(32.8)	428(33.5)	308(24.1)	124(9.7)
***χ***^***2***^		0.579	2.024	1.673	0.743
***P***		0.470	0.164	0.213	0.436

Data presented as a median and interquartile range; Continuous variables were compared using the Mann-Whitney test. Count data were expressed as rate (%) and analyzed by χ 2 test

*BMI* Body mass index, *P* Progesterone, *FSH* Follicle stimulating hormone, *LH* Luteinizing hormone, *E2* Estradiol

### The relationship between the distribution of the ABO blood type and the ovarian reserve with age less than 35 years

As shown in Table 3, in the present study, after excluding infertile women over 35 years, the relationship between the distribution of the ABO blood type and the ovarian reserve was analyzed by Chi-square test. The results showed that more patients with blood type O than other types in the DOR group (30.5%), while more patients with blood A than the other blood types in the non-DOR group (32.8%). Overall, blood type O was most prevalent in the DOR group (30.5%), followed by blood type A (28.9%), blood type B (28.3%), and blood type AB (12.3%). Meanwhile, blood type A was most prevalent in the non-DOR group (34.0%), followed by blood type O (32.8%), blood type B (34.0%), and blood type AB (9.5%). There were no significant differences in the proportions of blood types between the DOR and non-DOR groups (***P***_O_ = 0.552, ***P***_A_ = 0.177, ***P***_B_ = 0.193, ***P***_AB_ = 0.286, respectively). The above results suggest that blood group is not related to ovarian reserve capacity after excluding infertile women over 35 years. The detailed results are shown in Table 4.

**Table 4:** The distributions and comparisons of ABO blood type in patients with age were less than 35 years old in the DOR group and non-DOR. [(%)]

	n	ABO blood type			
		O	A	B	AB
DOR	**187**	**57(30.5)**	**54(28.9)**	**53(28.3)**	**23(12.3)**
non-DOR	**985**	**323(32.8)**	**335(34.0)**	**233(23.7)**	**94(9.5)**
***χ***^***2***^		**0.383**	**1.868**	**1.872**	**1.329**
***P***		**0.552**	**0.177**	**0.193**	**0.286**

Data presented as a median and interquartile range; Continuous variables were compared using the Mann-Whitney test. Count data were expressed as rate (%) and analyzed by χ 2 test

*BMI* Body mass index, *P* Progesterone, *FSH* Follicle stimulating hormone, *LH* Luteinizing hormone, *E2* Estradiol

## Discussion

This retrospective analysis used AMH and AFC values to determine normal ovarian reserve and DOR and concluded that there was no relationship between blood type and ovarian reserve in infertile women. Furthermore, after adjusting for age (< 35 years), history of EMS, and ovarian surgery, the correlation between blood type and ovarian reserve remained stable with no significant difference.

DOR, defined as a decreased quantity and quality of oocytes, affects nearly 10% of women seeking fertility treatment [32]. Multiple pathophysiologic factors affect ovarian reserve, including age, autoimmune conditions, ovarian surgery, chemotherapy, radiation, and genetics [33, 34]. Despite several studies explored the association between ABO blood type and ovarian reserve, the results were inconsistent. These conflicting findings may be due to racial variation between the study populations, because both blood type prevalence and ovarian reserve status differ among women of different races [35, 36]. For these reasons, only the Chinese Han population were included in the present study, and we ruled out that some other factors may have influenced the ovarian reserve.

In the current study, we found statistically significant differences in age, duration of infertility, BMI, FSH, FSH / LH elevated from the non-DOR group to the DOR group, and decreased levels of LH (*P* = 0.278) and progesterone (*P* = 0.002). Harzif et al. showed that ovarian reserve capacity decreases with age [37]. Xin et al. showed that age is a determinant of ovarian reserve [38]. The results were consistent with our study. Peng et al. showed that although there were differences in the duration of infertility, the differences between the pregnancy and non-pregnancy groups were not statistically significant [39]. The duration of infertility may affect ovarian reserve, but the exact mechanism needs to be further investigated. Age, duration of infertility, BMI, FSH and FSH / LH were negatively correlated with AMH while the P was positively correlated in our study. This difference was noticeable and statistically significant. Similar conclusions have been reached in other studies [40–42].

Moreover, we found that the most common ABO blood types in the DOR group were O (*n* = 143, 34.8%) and A (*n* = 122, 29.7%), while A (*n* = 428, 33.5%) and O (*n* = 419, 32.8%) were most frequent in the non-DOR group, respectively. Different gene expressions led to possible causes because genes determine the ABO blood type. ABO was the first blood group system discovered in humans and its identity is encoded by the ABO gene [43]. The gene that determines the ABO blood group is located on chromosome 9. The ABO gene, located on chromosome 9, consists of seven exons that encode the glycosyltransferase, determining the ABO blood group type [44]. Human blood groups are genetically characterized, and the gene group antigens that determine the blood group are aggrecan and controlled by three alleles of ABO [45]. Blood type O may be a risk factor for ovarian function, while blood type A is a protective factor. Further studies are needed to demonstrate the findings suggested in this analysis.

In our study, we found that the most common ABO blood types were O [*n* = 57, 30.5%] and A (*n* = 54, 28.9%) in the DOR group, while A [*n* = 335, 34.0%] and O (*n* = 323, 32.8%) accounted for the most in the non-DOR group in women < 35 years, respectively. Li et al. found that age was an independent factor affecting ovarian function, especially in those > 40 years, ovarian function decreased more than those < 40 years (28.4 vs. 65.2%) [46]. Yu et al. found that women over 35 had decreased ovarian function [47]. After adjusting for age, we still found that type O blood accounted for the highest proportion in the DOR group [57 (30.5) %], and type A blood accounted for the highest proportion in the non-DOR group [335 (34.0%)]. Type A blood is still a protective factor for ovarian function, while type O blood is a risk factor for ovarian function. Accordingly, we are supposed to speculate that age did not affect the blood type distribution between DOR group and non-DOR group, and there was still no potential difference between DOR group and non-DOR group in our study. Mu et al. found that ABO blood type was associated with ovarian reserve in Chinese women with subfertility [22]. A meta-analysis showed that there was no significant difference in the incidence of DOR between blood group A/B/AB/non-O and blood group O [48]. Therefore, more clinical studies are needed to prove this deduction. So far, there is no clear evidence that blood type is directly related to ovarian reserve function. Our results indicated that blood type does not constitute an ovarian reserve risk or protective factor. Therefore, blood type should not be considered when assessing ovarian reserve. However, our results require further studies to be validated.

In conclusion, a growing number of studies have confirmed the existence of a relationship between ABO blood group and ovarian reserve function. However, the results vary depending on the study design, population, sample size, ovarian function predictors and specific cut-off values. Therefore, broader sample size prospective studies are needed to confirm whether blood type independently affects ovarian reserve function and to elucidate the mechanisms through more in-depth, even molecular and genetic studies.

There were several strengths of our study. This study is the first to examine the region’s blood group and ovarian reserve in infertile population. This allows us to better understand the situation related to infertility in this region. A relatively large number of patients were included in this study compared to other clinical follow-ups, allowing for highly detailed information on comorbidities, hospitalization parameters and treatments, which contributed to the validity of this study. Age factors that may have influenced the results were excluded. Nevertheless, there are some potential limitations of this study. This study is a retrospective single-center analysis. Although all patients at our reproductive center who underwent assisted reproductive technologies (ART) during this period were included, the number of patients was relatively small. Our study was conducted in infertile women and is not representative of women with normal fertility. The participants in our study were solely from the Chinese Han ethic group and may not be representative of other ethnical groups. The relationship between ABO blood group and ovarian reserve was not elucidated.

## Conclusions

It was found that AMH was correlated with age, infertility duration, BMI, FSH, FSH/LH, and P. Furthermore, AFC was correlated with age, FSH, and FSH/LH. However, this study found no significant correlation between ovarian reserve and ABO blood group in infertile women. Whether blood type independently affects ovarian reserve function requires a broader sample size prospective study to clarify the mechanism by more in-depth or even molecular and genetic studies.

## Data Availability

Data in the article can be found in the department of Reproductive Medicine Center, the Affiliated Hospital of Southwest Medical University electronic medical record system.
